# Curcumenol Targeting YWHAG Inhibits the Pentose Phosphate Pathway and Enhances Antitumor Effects of Cisplatin

**DOI:** 10.1155/2022/3988916

**Published:** 2022-06-26

**Authors:** Zhijie Mao, Liyan Zhong, Xiaodan Zhuang, Haoen Liu, Yan Peng

**Affiliations:** ^1^ChangZhou Wujin People's Hospital, Changzhou 213017, Jiangsu, China; ^2^Wujin Hospital Affiliated with Jiangsu University, Changzhou 213017, Jiangsu, China; ^3^The Wujin Clinical College of Xuzhou Medical University, Changzhou 213017, Jiangsu, China

## Abstract

**Objective:**

Cervical cancer is a common cancer in women. The drug resistance of chemotherapeutic agents has always been an urgent problem to be solved in clinics. The purpose of this study was to determine the role of tyrosine 3-monooxygenase/tryptophan 5-monooxygenase activation protein gamma polypeptide (YWHAG) in cervical cancer and explore the effect of *Curcuma* on cervical cancer and its possible mechanism.

**Methods:**

YWHAG expression in cervical cancer was confirmed using The Cancer Genome Atlas (TCGA) database. Then, the effects of YWHAG on the proliferation and invasion of HeLa and C33A cervical cancer cells were detected by the cell counting kit-8 (CCK-8) and transwell assay. The relationship between YWHAG and the pentose phosphorylation pathway was further studied. CCK-8, Edu, and quantitative real-time polymerase chain reaction were used to confirm that *Curcuma* inhibited the sensitivity of YWHAG to cisplatin chemotherapy and to detect the expression of apoptosis-related proteins.

**Results:**

YWHAG was highly expressed in cervical cancer and was associated with poor prognosis. The proliferation and invasion abilities of HeLa and C33A cells decreased after YWHAG knockout. The TCGA database of cervical cancer showed a positive correlation between YWHAG and hypoxia-inducible factor-1 subunit alpha (HIF-1*α*) expression. YWHAG expression increased with HIF-1*α* overexpression. YWHAG knockdown reduced the protein expression in the pentose phosphorylation pathway. Curcumenol inhibited YWHAG expression. Compared with cisplatin alone, curcumenol combined with cisplatin can reduce cell proliferation and invasion and reduce matrix metalloproteinase (MMP) 2 and MMP9 expression. It can also increase apoptosis, decrease B cell lymphoma 2 (Bcl-2) expression, and increase the expression of Bcl-2 antagonist X, caspase-3, and polyadenosine diphosphate-ribose polymerase.

**Conclusion:**

YWHAG can interact with HIF-1*α* to affect the proliferation and invasion of cervical cancer cells. YWHAG knockout can reduce the expression of pentose phosphorylation pathway-related proteins. Curcumenol can enhance cisplatin to inhibit cancer cell proliferation, migration, and invasion and promote tumor cell apoptosis. The combination of drugs may promote the apoptosis of cervical cancer cells through the YWHAG pathway.

## 1. Introduction

Cervical cancer, the second most common cancer in women after breast cancer, is the most common gynecological cancer in developing countries [1, 2]. Patients with early stage cervical cancer and locally advanced cervical cancer can receive conventional treatment, including surgery, chemotherapy, and radiation. However, metastatic breast cancer has no standard treatment because of its heterogeneity, and its median survival is only 8–13 months [3]. Cisplatin is a small-molecule platinum compound and is the most effective anticancer drug in the treatment of advanced/recurrent cervical cancer [4]. Cisplatin covalently binds the DNA of cancer cells to form DNA–cisplatin complexes, which then induces DNA damage and leads to cancer cell apoptosis and death [5]. Cisplatin combined with paclitaxel is the standard chemotherapy regimen for the treatment of recurrent or metastatic breast cancer, but resistance to cisplatin affects its use in clinical practice [4]. The mechanism of cisplatin resistance is related to the decreased accumulation of platinum compounds, increased repair of DNA damage, apoptosis inactivation, and activation of epithelial-mesenchymal transformation (EMT). Among them, apoptosis induced by cisplatin is very important for its therapeutic effect. Compared with sensitive cells, cisplatin-resistant HeLa cells show lower apoptosis and lower expression of Bcl-2 and p-Bad [6]. In addition, SiHa cells are more resistant than HeLa cells [7]. Based on the mechanism of cisplatin resistance, finding targets is crucial to improve its sensitivity.

Tyrosine 3-monooxygenase/tryptophan 5-monooxygenase activation protein gamma polypeptide (YWHAG, 14-3-3*γ*) is a highly conserved protein that mediates cell signaling by binding to phosphorus-containing proteins. Some reports suggested that miRNA is involved in regulating YWHA to affect tumor progression. miR-181b-3p promotes EMT in breast cancer cells by directly targeting YWHAG [8]. miR-217 affects glioblastoma progression by targeting YWHAG and regulating MDM4/p53 signal transduction, which is expected to be a therapeutic target or diagnostic biomarker for glioblastoma [9]. Similar results were observed in osteosarcoma, where miR-222 inhibits cell proliferation and invasion by downregulating YWHAG [10]. Genetic variations of chromosomes also affect YWHAG expression. The genetic variation of 15q13.3 and 7q11.23 can cause gastric cancer progression by regulating the function of YWHAG [11]. Whether YWHAG also plays a role in cervical cancer, it still needs further study.

Hypoxia-inducible factor-1 (HIF-1*α*) is a heterodimer whose expression is highly regulated and depends on the rate of prealbumin synthesis and protein degradation. Su et al. found that miR-200 promotes the proliferation of cervical cancer cells by regulating the HIF-1*α*/VEGF signaling pathway [12]. Some studies also found that HIF-1*α* is remarkably downregulated in cervical cancer tissues after chemotherapy compared with before chemotherapy, suggesting that HIF-1*α* can be used as a potential biomarker to predict the sensitivity of cisplatin chemotherapy in cervical cancer [13].

Curcumenol showed certain antitumor effects in malignant epithelial tumors, such as cervical cancer, cervical cancer, breast cancer, and digestive tract cancers [14]. However, few studies have been conducted on the mechanism of curcumenol against cervical cancer, and the combination of curcumenol and platinum drugs in the treatment of cervical cancer has not been reported.

The purpose of this study was to investigate the effects of curcumenol on YWHAG and its mechanism on cervical cancer cells and cisplatin chemotherapy resistance to provide a new approach for the molecular diagnosis and treatment of cervical cancer.

## 2. Methods

### 2.1. Cell Culture

Human cervical cancer cell lines (HeLa and C33A) were purchased from the American Type Culture Collection. The cells were cultured in an incubator with 5% CO_2_ at 37 °C in RPMI 1640 medium (Hyclone, USA) supplemented with 10% fetal bovine serum (Gibco, USA), 100 U/mL penicillin, and 100 ug/mL streptomycin (Sigma, St. Louis, MO, USA). The cell culture medium was changed every other day, and cell passage was carried out according to the cell growth density in the culture dish. Cells at the logarithmic growth phase were selected for the cell function experiments.

### 2.2. Cell Transfection

YWHAG-silencing RNA (si-YWHAG) and corresponding controls were synthesized from RiboBio (Guangzhou, China). The human cervical cancer cells were inoculated into 96-well plates at a density of 2 × 10^3^/plate. si-YWHAG and its blank control were added to Lipofectamine 2000 transfection reagent and gently added to the well covered with cells. The transfection reagent complex was evenly mixed in the cell suspension. The cells were incubated in a constant-temperature incubator for 24 h. The cell transfection supernatant was poured out and replaced with Dulbecco's modified Eagle's medium with 10% FBS for further culture. Protein expression was detected after 3-4 days of culture.

### 2.3. Cell Counting Kit-8 (CCK-8) Assay

The human cervical cancer cells were seeded into a 96-well plate at 1 × 10^6^/mL and cultured in an incubator at 37°C with 5% CO_2_. After the cells adhered to the wall, CCK-8 with a medium volume of 10/1 was added. Then, the cells were placed in the incubator, and culturing was continued for 4 h. The specific time was determined by the color of the culture medium. The cells were detected when the color turned orange. The 96-well plate was placed in a microplate reader, and the absorbance value was read at 450 nm.

### 2.4. Transwell Assay

A 100 *μ*L of Matrigel was added into the upper transwell chamber and polymerized into a gel at 37°C for 30 min. The cells were seeded in the upper chamber of the transwell at a density of 5 × 10^4^, and a medium containing 10% FBS was added. FBS was added to the lower chamber. The cells were placed at 37°C with 5% CO_2_ and incubated for 24 h. A cotton swab was used to gently wipe off the cells on the surface of the lower chamber, and cells in the upper chamber were stained with 0.1% crystal violet. The number of stained cells was counted under a microscope.

### 2.5. Bioinformatics Analysis

All analyzed data came from The Cancer Genome Atlas (TCGA) database. The key cancer-promoting genes in cervical cancer were analyzed through the Protein Atlas website (https://www.proteinatlas.org/). The effect of YWHAG on the prognosis of patients with cervical cancer was analyzed on the OncoLnc website (http://www.oncolnc.org/). The interaction between YWHAG and HIF-1*α* was completed through the Gene Expression Profiling Interactive Analysis website (http://gepia.cancer-pku.cn/).

### 2.6. RNA Extraction and Quantitative Real‐Time Polymerase Chain Reaction (qRT-PCR) Detection

TRIzol was used to extract total RNA from human cervical cancer cells. RNA samples were reverse-transcribed into cDNA using PrimeScript™ RT Master Mix (TakaRa, Japan). qRT-PCR was prepared using 2 × SYBR Green according to the manufacturer's instructions. The reaction condition was 95°C for 5 min and then forty cycles of 95°C for 30 s, 58°C for 30 s, and 72°C for 30 s. After the reaction was completed, the cyclic threshold for each reaction was calculated, and the protein content was calculated using the 2^−ΔΔCt^ method. The primer sequences for qPCR analysis are given Table 1.

### 2.7. Western Blot

Total protein extraction was performed. The protein samples were separated by sodium dodecyl sulfate-polyacrylamide gel electrophoresis. The protein was then transferred to a polyvinylidene fluoride membrane (PVDF) and blocked with 5% skim milk for 2 h. The PVDF membrane containing proteins was incubated with primary antibodies (anti-YWHAG, 1 : 500, Invitrogen) at 4°C overnight and then incubated with the secondary antibody at room temperature for 1 h. Western blot was performed in an enhanced chemiluminescence system.

### 2.8. Immunofluorescence Costaining Assay

The cells were seeded on the cell slide of the 24-well plate. After cell adherence, the cells were fixed with 4% paraformaldehyde for 15 min. Triton X-100 was then used for permeation for 10 min. Then, the cells were sealed with 5% BSA for 30 min. The primary antibody was added and incubated overnight at 4°C in a humid environment (rabbit-derived polyclonal antibody YWHAG, 1 : 200, Invitrogen; mouse-derived monoclonal antibody HIF-1*α*, 1 : 100, Invitrogen). On the next day, goat anti-rabbit and goat anti-mouse horse radish peroxidase secondary antibodies (Invitrogen) labeled with fluorescein isothiocyanate were added and incubated at room temperature for 2 h. In addition, 4′,6-diamidino-2-phenylindole sealing was used. The intensities of YWHAG and HIF-1*α* in each group were observed under a fluorescence microscope. Fluorescence intensity was quantified by the ImageJ software.

### 2.9. Metabolite Detection of the Pentose Phosphate Pathway (PPP)

The glucose and lactic acid produced by the cells were consumed, and then, the medium was changed and incubated for another 24 h. Glucose levels in the medium were determined using a glucose colorimetric kit (BioVision). Total protein content was determined by a bicinchoninic acid protein determination kit (Beyotime). After cell lysis, D-sedoheptulose-1,7-biphosphate, deoxyribose-phosphate, fructose 1, 6-biphosphate, xylulose 5-phosphate, octulose-1, 8-biphosphate, and ribose-5-phosphate enzyme activities and intracellular NADPH level were detected by a detection kit (Yuanye).

### 2.10. Terminal Deoxynucleotidyl Transferase Biotin-dUTP Nick End Labeling (TUNEL) Assay

The cells were seeded on the cell slide of a 24-well plate. The cell slides were stained according to a TUNEL kit. Apoptotic cells were counted in the stained cell slides under a fluorescence microscope (543 nm excitation wavelength and 571 nm emission wavelength).

### 2.11. Statistical Analysis

All data were analyzed by SPSS 23.0 for counting data, and the *χ*^2^ test was used for comparison between the groups. The measurement data are expressed as mean ± standard deviation. The two independent sample *t*-test was used for comparison between the two groups, and the nonparametric rank-sum test was used for data that did not meet the homogeneity of variance. *P* < 0.05 was considered statistically significant.

## 3. Results

### 3.1. YWHAG as a Key Oncogenic Gene in Cervical Cancer

The analysis of the TCGA database showed that YWHAG was highly expressed in a variety of tumors, including cervical cancer (Figure 1(a)). The effect of YWHAG on the prognosis of patients with cervical cancer was analyzed, and the results showed that high YWHAG expression in patients with cervical cancer was statistically significant (*P* < 0.05, Figure 1(b)).

### 3.2. Low YWHAG Expression Inhibits the Proliferation, Invasion, and Migration of Cervical Cancer Cells

YWHAG in cervical cancer cell lines was knocked out, and its expression was detected by qPCR as shown in Figure 2(a). The knockout efficiencies of YWHAG-KD1 and YWHAG-KD2 in HeLa cells were 0.824 and 0.832, respectively, and in C33A cells were 0.789 and 0.841, respectively, . CCK-8 was used to detect the proliferation of cells with YWHAG knockout. The results showed that compared with the NC group, the proliferation ability of the cervical cancer cells was weakened after YWHAG knockout (Figures 2(b) and 2(c)). Cell invasiveness was detected by transwell assay. Experimental results suggested that compared with the NC group, the invasion ability of cells in the YWHAG knockout group was weakened (Figures 2(d) and 2(e)). Therefore, low YWHAG expression can inhibit the proliferation and invasion of cervical cancer cells.

### 3.3. YWHAG Interacts with HIF-1*α* in Cervical Cancer

Cervical cancer data from TCGA were analyzed, and the correlation between YWHAG and HIF-1*α* in cervical cancer samples was measured using a microarray platform to investigate the proteins interacting with YWHAG that inhibit the proliferation of cervical cancer cells. Pearson' correlation test showed that YWHAG was positively correlated with HIF-1*α* expression (Figure 3(a)). Then, Western blot was used to detect their relationship. The results showed that YWHAG expression upregulated after HIF-1*α* overexpression (Figure 3(b)). Moreover, the expression of the two proteins in cells was observed by immunofluorescence assay. The results indicated that YWHAG and HIF-1*α* were coexpressed in the cytoplasm (Figure 3(c)). In sum, YWHAG interacted and was positively correlated with HIF-1*α* in cervical cancer cells.

### 3.4. YWHAG Is Associated with the PPP in Cervical Cancer

Changes in metabolites of the PPP, including D-sedoheptulose-1,7-biphosphate, deoxyribose-phosphate, fructose 1, 6-biphosphate, xylulose 5-phosphate, octulose-1,8-biphosphate, and ribose-5-phosphate, and the effect of glucose uptake ability of cells were analyzed to study the pathway of YWHAG affecting cervical cancer. The results showed that after YWHAG knockout, the expression levels of the above proteins decreased, and the glucose uptake was reduced as shown in Figures 4(a)–4(g). In conclusion, YWHAG can inhibit the PPP in cervical cancer cells and reduce glucose uptake.

### 3.5. Curcumenol Inhibits YWHAG and Increases the Sensitivity of Cervical Cancer Cells to Chemotherapy

Figure 5(a) shows that curcumenol inhibited YWHAG expression in a dose-dependent manner. Cisplatin is a common drug in chemotherapy, and drug resistance is now a common problem. Changes in its sensitivity were studied to verify the effect of curcumenol on cisplatin chemotherapy. The results suggested that the proliferation and invasion abilities of the curcumenol + cisplatin group were reduced compared with that of the cisplatin group. The expression levels of matrix metalloproteinase (MMP) 2 and MMP9 also decreased (Figures 5(b)–5(e)).

### 3.6. Curcumenol Treatment Increased Cisplatin-Induced Apoptosis

The effect of curcumenol on sensitivity to cisplatin chemotherapy was determined. We further studied the way in which curcumenol increases the sensitivity of cisplatin by apoptosis assay and the expression of related apoptotic proteins. TUNEL experiment was performed to determine its effect on apoptosis. The results showed that compared with the cisplatin group, the curcumenol + cisplatin group could increase the apoptosis rate of cells (Figure 6(a)). Moreover, we detected the expression of apoptosis-related proteins, including B cell lymphoma 2 (Bcl-2), Bcl-2 antagonist X (Bax), caspase-3, and polyadenosine diphosphate-ribose polymerase (PARP). The results indicated that curcumenol could increase the expression levels of Bax, caspase-3, and PARP and decrease the expression of Bcl-2 (Figures 6(b)–6(e)). Therefore, curcumenol can increase the sensitivity of cisplatin chemotherapy and then induce cell apoptosis.

## 4. Discussion

The results of this study showed that YWHAG was highly expressed in cervical cancer cells, and patients with high YWHAG expression had a poor prognosis. In vitro function experiment showed that the proliferation and invasion abilities of YWHAG-overexpressing cells were inhibited. In addition, the effect of YWHAG on cervical cancer cells is exerted through its interaction with HIF-1*α*, which then affects the PPP. Curcumenol can inhibit YWHAG, increase the sensitivity of cisplatin chemotherapy, and increase cisplatin-induced apoptosis.

YWHAG is a 14-3-3*γ*, a member of the 14-3-3 family in mammals. 14-3-3 proteins are involved in regulating a variety of cellular processes, including the cell cycle, protein transport, cell survival, and apoptosis [15]. The 14-3-3 subtype, including YWHAG, can bind to Snail and influence the progress of EMT [16, 17]. YWHAG has different effects in different tumors. Pritsana et al. also showed that YWHAG knockout could reduce ETM-associated proteins, MMP2 and MPP9, in nonsmall cell lung cancer [18]. In breast cancer, miR-181b-3p promotes EMT of breast cancer cells by targeting YWHAG [8]. However, YWHAG acts as a tumor suppressor gene, and miR-217 promotes cell proliferation and invasion by targeting tumor suppressor genes in glioblastoma [9]. As one of the subtypes of the 14-3-3*β* protein, circSMARCA5 has been found to inhibit the proliferation and invasion of cervical cancer cells by inhibiting the binding of SND1 and YWHAB [19]. We first analyzed relevant data in TCGA to clarify the role of YWHAG in cervical cancer. The results showed that YWHAG was highly expressed in cervical cancer cells, and the survival of these patients was shorter. YWHAG knockout resulted in the inhibition of the proliferation and invasion of cervical cancer cells. Consistent with previous studies, YWHAG, as an oncogenic gene, promotes the viability of cervical cancer cells.

Chemotherapy, as the first-line cancer treatment, still plays an important role in cancer treatment. However, tumor cells affect the sensitivity of chemotherapy through a variety of intrinsic factors or mechanisms of acquired drug resistance [20–22]. Resistance mechanisms, including drug metabolism changes, drug transport disorders, and changes in target protein receptors, lead to drug resistance [23, 24]. Cisplatin, the most widely used cancer drug, is used to treat a variety of cancers, including ovarian cancer, bladder cancer, gastric cancer, and nonsmall cell lung cancer [25]. Although cisplatin's cytotoxicity can affect the kidneys, peripheral nerves, and ears, the main limitation of its clinical utility is its high resistance rate [26]. At present, the mechanisms of cisplatin resistance are divided into three aspects: changes in DNA repair, intracellular drug accumulation, and drug inactivation in cell solutes [27–30]. Low levels of drug resistance are associated with changes in DNA repair. Moderate resistance was associated with reduced intracellular cisplatin accumulation. The cytoplasmic inactivation of cisplatin is the main mechanism at high resistance levels [31]. In drug-resistant tumor cells, all three mechanisms often coexist. Therefore, finding pathways that can increase the sensitivity of cisplatin chemotherapy is essential. Li et al. studied the potential markers of cisplatin-induced endothelial damage in patients with cancer and found that *PARP1*, as a key gene of endothelial damage, plays a role in DNA damage repair induced by cisplatin by regulating YWHAB [32]. As one of the similar subtypes, YWHAG may affect the DNA damage repair process induced by cisplatin to affect cell apoptosis and thus increase the sensitivity of chemotherapy. Our results also indicated that low YWHAG levels can increase cisplatin-induced apoptosis. Therefore, YWHAG may serve as a sensitive target of cisplatin chemotherapy resistance and make contributions to overcoming cisplatin resistance in the future.

HIF-1*α* has been identified as an important transcription factor involved in tumorigenesis and tumor development by regulating the expression of genes related to angiogenesis, tumor metastasis, cell proliferation, and chemoradiotherapy resistance [33, 34]. The role of HIF-1*α* has also been found in cervical cancer [35, 36]. HIF-1*α* regulates tumor angiogenesis by regulating various angiogenic factors under hypoxia [37]. Hypoxia is a common feature in cervical cancer microenvironment, in which HIF-1*α* is accumulated. miR-200 promotes the proliferation of cervical cancer cells by regulating the HIF-1*α*/VEGF signaling pathway [38]. miR-200 promotes the proliferation of cervical cancer cells by regulating the HIF-1*α*/VEGF signaling pathway [12]. Moreover, as a hypoxia-induced transcription factor, HIF-1*α* may also protect cervical cancer cells from radiation-induced apoptosis through various mechanisms. Song et al. found that miR-21 affects the HIF-1*α* expression through a positive feedback loop with the PTEN/Akt/HIF-1*α* pathway, which reduces the autophagy of cervical cancer cells and reduces their radiation resistance [39]. As a key gene in the feedback regulatory loop, HIF-1*α* affects the sensitivity of cervical cancer cells to chemotherapy. In this study, the expression levels of YWHAG and HIF-1*α* were positively correlated and interacted with each other. We speculated that the increased sensitivity of YWHAG to cisplatin is caused by its interaction with HIF-1*α*.

Intracellular glucose is metabolized by glycolysis or obtained by pentose phosphorylation. Rapidly growing and dividing cancer cells absorb excess glucose and break it down by aerobic glycolysis [40]. This metabolic change is a hallmark of cancer cells [41]. In the present study, the expression of metabolites in the PPP decreased in cervical cancer cells after YWHAG knockout, suggesting that YWHAG is a key gene in the pentose phosphorylation process, and its effect on cervical cancer cells may be realized through this pathway.

Curcumenol has a variety of pharmacological and biological activities, including antitumor activity, treatment of nerve and mental diseases, and antiliver fibrosis [42–44]. Studies confirmed that curcumenol has antitumor effects on gastric cancer, colorectal cancer, and breast cancer [45, 46]. Studies showed that curcumenol can inhibit the growth and metastasis of lung adenocarcinoma by inhibiting the activation of the PI3K/AKT and Wnt/*β*-catenin pathways [47]. Curcumenol also inhibits the drug resistance of lung cancer to tumor necrosis factor-related apoptosis-inducing ligands by directly targeting the regulation of quinone oxidoreductase 2 [48]. However, the regulatory mechanism of curcumenol on cervical cancer has not been fully elucidated.

In this study, curcumenol inhibited the proliferation and invasion of HeLa and C33A cells and promoted the apoptosis of cervical cancer cells by targeting YWHAG. Curcumenol has an antitumor effect and can be used as a sensitizer of first-line chemotherapy drugs. Studies reported that curcumenol can increase the sensitivity of lung cancer cells to cefazolin sodium chemotherapy [49] and can inhibit the proliferation of colon cancer cells through the PI3K/AKT pathway to play an antitumor effect [50]. Circular RNA circ_0020123 regulated THBS2 by sponging miR-590-5p to promote cell proliferation and migration and inhibit cell apoptosis in NSCLC cells [51]. In the present study, curcumenol enhanced the inhibitory ability of cisplatin on the proliferation, migration, and invasion of cervical cancer cells and promoted the apoptosis of cervical cancer cells.

This study still has many deficiencies. First, the factors affecting cervical cancer were determined only by in vitro experiments. Furthermore, in vivo experiments are needed for further study. Second, the downstream pathway of YWHAG–HIF-1*α* interaction that regulates the radiotherapy sensitivity of cervical cancer needs to be further studied to improve the research results. Third, the analysis of YWHAG is one-way. More experiments are needed to prove the correlation between the research indicators.

Overall, this study found that curcumenol inhibited YWHAG and increased apoptosis by increasing the sensitivity of cisplatin chemotherapy. It provides a new target for the treatment and diagnosis of cervical cancer in the future.

## 5. Conclusion

In conclusion, this study found that low YWHAG expression is remarkably associated with the poor prognosis of patients with cervical cancer. Curcumenol inhibited YWHAG and increased the sensitivity of cisplatin chemotherapy and cancer cell apoptosis. This effect may be achieved through the PPP.

## Figures and Tables

**Figure 1:** YWHAG is a key oncogenic gene in cervical cancer. (a) TCGA data showing that YWHAG was highly expressed in a variety of tumors. (b) TCGA data showing that cervical cancer patients with high expression of YWHAG had a poor prognosis. TCGA, The Cancer Genome Atlas.

**Figure 2:** YWHAG gene knockdown (KD) inhibits proliferation, invasion, and migration of cervical cancer. PCR assay used to detect YWHAG knockdown (KD) in HeLa and C33A (a). CCK-8 detected the proliferation of HeLa (b) and C33A (c). The invasiveness of HeLa (d) and C33A (e) detected by transwell assay. qRT-PCR, quantitative real-time PCR. ^*∗∗*^*P* < 0.01. Scale = 200 *μ*m.

**Figure 3:** YWHAG interacts with HIF-1*α* in cervical cancer. (a) TCGA cervical cancer data analysis, correlation of YWHAG, and HIF-1*α* expression in cervical cancer samples measured by microarray platform; Western blotting was used to detect the expression of YWHAG in HeLa (b). The expression positions of YWHAG and HIF-1*α* in HeLa (c) detected by immunofluorescence. TCGA, The Cancer Genome Atlas. ^*∗∗*^*P* < 0.01. Scale = 5 *μ*m.

**Figure 4:** YWHAG is associated with the pentose phosphate pathway (PPP) in cervical cancer. Metabolites of the pentose phosphate pathway were detected in HeLa and C33A cells, including D-sedoheptulose-1,7-biphosphate (a), deoxyribose-phosphate (b), fructose 1, 6-biphosphate (c), xylulose 5-phosphate (d), octulose-1, 8-biphosphate (e), and ribose-5-phosphate (f). (g) Glucose uptake capacity of HeLa and C33A cells. ^*∗*^*P* < 0.05, ^*∗∗*^*P* < 0.01.

**Figure 5:** Curcumenol increased chemotherapy sensitivity of cisplatin by inhibiting YWHAG. (a) The expression of YWHAG detected by qRT-PCR. (b) The proliferation of C33A cells detected by CCK-8 assay. (c) Transwell assay used to detect the invasion ability of C33A cells. (d) The expression of MMP2 in C33A cells detected by qRT-PCR assay. (e) Changes of MMP2 expression in C33A cells detected by qRT-PCR assay. ^*∗*^*P* < 0.05, ^*∗∗*^*P* < 0.01, ^*∗∗∗*^*P* < 0.001. Scale = 200 *μ*m.

**Figure 6:** Curcumenol treated increase cisplatin-induced apoptosis. (a) Apoptosis of C33A cells detected by TUNEL assay. (b) The expression level of Bax in C33A cells detected by qRT-PCR assay. (c) The expression level of Bcl-2 in C33A cells detected by qRT-PCR assay. (d) qRT-PCR assay used to detect the expression of caspase-3 in C33A cells. (e) The expression level of PARP in C33A cells detected by qRT-PCR assay. qRT-PCR, quantitative real-time PCR. ^*∗*^*P* < 0.05, ^*∗∗*^*P* < 0.01, ^*∗∗∗*^*P* < 0.001.

**Table 1:** Primer sequences for qRT-PCR.

	Sequences (5′–3′)	
	Forward	Reverse
YWHAG	GCCGTATGTCAGGATGT	GCCAGGTAGCGGTAAT
MMP2	CACCATGGGTTCTGGTCA	GGGGACTGGGATACAGCCTT
MMP9	TGAGCAGCTGCAAACGACTA	CACGAACTGCCTGGTACTGT
Bax	TCCACCAAGAAGCTGAGCGAG	GTCCAGCCCATGATGGTTCT
Bcl-2	TTCTTTGAGTTCGGTGGGGTC	TGCATATTTGTTTGGGGCAGG
Caspase-3	TTAATAAAGGTATCCATGGA	TTAGTGATAAAAATAGAGTT
PARP	GATGTCACTGCCTGGACCAA	GCTTCGTCCTTGTTCTGGGA
GAPDH	ACGGCAAGTTCAACGGCACAG	GAAGACGCCAGTAGACTCCACGAC

## Data Availability

The data used to support the findings of this study are available from the corresponding author upon request.
